# Chemoradiotherapy and Increased Prescription Dose in Esophageal Squamous Cell Cancer: A Retrospective Study

**DOI:** 10.1155/2021/3834040

**Published:** 2021-02-08

**Authors:** Xiaofen Pan, Mingchu Liao, Hongmei Ma, Xiaobing Jiang, Hanwen Huang, Min Wei, Qun Li

**Affiliations:** ^1^Department of Oncology, The Seventh Affiliated Hospital, Sun Yat-sen University, Shenzhen, China; ^2^Department of Medical Oncology, The First Affiliated Hospital of University of South China, Hengyang, China; ^3^Department of Medical Oncology, The First People's Hospital of Chengdu, Chengdu, China; ^4^Department of Neurosurgery/Neuro-oncology, Sun Yat-sen University Cancer Center, State Key Laboratory of Oncology in South China, Collaborative Innovation Center for Cancer Medicine, Guangzhou, China; ^5^Department of Oncology, Yunfu People's Hospital of Guangdong, Yunfu, China; ^6^Department of Radiation Oncology, Sun Yat-sen University Cancer Center, State Key Laboratory of Oncology in South China, Collaborative Innovation Center for Cancer Medicine, Guangzhou, China

## Abstract

To analyze the outcomes and adverse events of patients with esophageal squamous cell carcinoma (ESCC) treated with definitive chemoradiation with modified radiotherapy volume and increased radiation dose. This was a retrospective analysis of patients with ESCC treated with definitive chemoradiotherapy at the Sun Yat-sen University Cancer Center (02/2015 to 02/2017). The dose to the planning gross tumor volume (PGTV) and planning clinical tumor volume (PTV1) was 66-68 Gy (2.0-2.2 Gy/fraction). The dose to the planning regional lymph node drainage area volume (PTV2) was 46 Gy (2.0 Gy/fraction). Treatment response, adverse events, progression-free survival (PFS), overall survival (OS), and locoregional failure-free survival (LRFFS) were analyzed. Twenty-six patients were included. The median follow-up was 31 (range, 4.3-51.3) months. Sixteen (61.5%) patients had a complete response, and four (15.4%) achieved a partial response. The objective response rate was 76.9%, and the disease control rate was 80.8%. The median PFS and OS were not achieved. The 4-year PFS was 63.9%, and the 4-year OS was 71.0%. Grade 1-2 and 3-4 radiation-related esophagitis was observed in 15 (57.7%) and one (4.5%) patients, respectively. Grade 1-2 and 3-4 radiation-related pneumonitis was observed in 12 (46.2%) and one (4.5%) patients, respectively. No patients developed radiation-related heart or skin damage. The modified target volume definition and increased dose of definitive radiotherapy combined with chemotherapy in patients with ESCC had low toxicity and might improve survival, but additional trials are necessary to prove the superiority of this strategy.

## 1. Introduction

Esophageal cancer is the eighth leading cause of cancer death in the world [1]. Esophageal squamous cell carcinoma (ESCC) and adenocarcinoma are the two common subtypes of esophageal cancer. In East Asia, ESCC is the most common type of esophageal cancer, while adenocarcinoma is more prevalent in western countries [2]. These two types differ in pathogenesis, prognosis, and tumor biology [3].

For early-stage esophageal cancer, surgery remains the standard therapy, but the patients still have 3-5-year survival rates of 5%-32% [4]. The combination of chemotherapy and radiotherapy improves local control and overall survival (OS) rates in medically fit populations [5]. In Europe and North America, 50.4 Gy is the standard dose for a patient undergoing definitive chemoradiation, based on the RTOG 90-12 and INT0123 trials [6]. Even though dose escalation showed no improvement to local control and OS, 60.0 Gy remains a commonly used dose in Asian countries [7], where ESCC is more common than in western countries where most trials were conducted [2]. A pooled analysis showed that the median progression-free survival (PFS) ranged from 7.4 to 12.0 months, and OS ranged from 9.0 to 34.0 months; the 1-, 2-, and 3-year pooled OS rates were 57%, 39%, and 40%, respectively [8].

Intensity-modulated radiation therapy (IMRT) has the advantage of limiting the radiation dose to organs at risk without reducing the dose delivered to the tumor [9]. IMRT has a benefit in decreasing pulmonary complications, but IMRT failed to show a cancer-specific survival over three-dimensional radiation (3DCRT) when using the current standard radiation therapy doses [10]. A study from the MD Anderson Cancer Center showed the failure patterns in patients treated by IMRT based on modern-day radiation treatment volumes [9]. The study indicated that 50% of patients had a local failure, while 48% had distant failures. Among the local failure cases, 90% were within the gross tumor volume (GTV), and 23% were within the clinical target volume (CTV) [9].

Therefore, the present study is aimed at analyzing the outcomes and adverse events of patients with ESCC treated with definitive chemoradiation with radiotherapy volume using modified GTV and CTV definitions and increased radiation dose.

## 2. Materials and Methods

### 2.1. Study Design and Patients

This was a retrospective analysis of patients with ESCC treated with definitive chemoradiotherapy at the Sun Yat-sen University Cancer Center between February 2015 and February 2017. This study was approved by the Ethics Committee of Sun Yat-sen University Cancer Center.

The inclusion criteria were as follows: (1) newly diagnosed and histologically proven ESCC [11], (2) ≥18 years of age at start therapy, (3) tumor was unsuitable for esophagectomy [12], (4) definitive chemoradiotherapy using IMRT, and (5) the target volume delineating method was modified according to the description in the radiation therapy part. The exclusion criteria were as follows: (1) history of other tumors, (2) treated for recurrent disease, (3) had distant metastasis (not including celiac or supraclavicular lymph nodes), or (4) received other 2D or 3D radiation therapy.

### 2.2. Radiation Therapy

The GTV includes the primary tumor (GTVt) and involved regional lymph nodes (GTVnd). The GTVt encompassed the primary tumor according to the CT scan and endoscopy. The volume of lymph nodes (GTVnd) encompassed lymph nodes in the drainage area shown by the CT scan, disregarding the diameters.

The CTV1 was defined as 3 cm above the proximal edge and 3 cm below the distal edge of the GTVt and 1-2 mm from the GTVt, outside the esophageal wall. The upper border of the CTV did not expand above the cricoid cartilage, and the lower border did not expand to the stomach unless a gross tumor was present at those levels. CTV2 for regional lymph nodal drainage area volumes was contoured according to the expert consensus contouring guidelines [13] (Figure 1).

The planning gross target volume (PGTVt) was defined as 0.5 cm from the GTVt in the superior-inferior directions and 0.5 cm in the right-left and the anteroposterior directions. The planning gross tumor volume of lymph nodes (PGTVnd) was defined as 0.5 cm from the GTVnd in the superior-inferior, right-left, and anteroposterior directions. The planning target volumes of CTV1 (PTV1) and CTV2 (PTV2) were defined as 0.5 cm from the CTV1 and CTV2 in the superior-inferior, right-left, and anteroposterior directions. The modified definitions of target volumes are shown in Table 1.

Radiation therapy was administered by IMRT technology with a total dose of 66-68 Gy delivered to the PGTVt and PGTVnd. The radiation therapy plan was designed as a one-stage or two-stage strategy. For the one-stage strategy, a dose of 44-46 Gy was delivered to the PTV2, and a dose of 66-68 Gy was delivered to the PGTVt, PGTVnd, and PTV1 by a simultaneously boost technology. For the two-stage strategy, a dose of 46 Gy was delivered to the PTV1, PTV2, PGTVt, and PGTVnd in conventional fractionation of 2.0 Gy/fraction in the first stage (stage A), and a dose of 20-22 Gy was delivered to the PGTVt, PGTVnd, and PTV1 in a fraction of 2.0-2.2 Gy/fraction in the second stage (stage B) right after stage A.

The lung V20 was defined as the proportion of lung volume receiving irradiation of ≥20 Gy to the total lung volume. In general, a one-stage design was first performed, and, then, the lung V20 was evaluated. If the lung V20 exceeded 30%, a two-stage design was performed to control the lung V20 to be within 30%. Later, it was found that the two-stage design of the patient's lung V20 was lower than the one-stage design, so the two-stage design was performed for patients later on. But regardless of the one- or two-stage design, the total radiation dose was the same.

Radiation therapies were performed by a radiation therapist with more than 30 years of experience in this field.

### 2.3. Chemotherapy

Some patients were scheduled for induction chemotherapy or concurrent chemotherapy. Chemotherapy consisted of paclitaxel/nedaplatin, paclitaxel/5-fluorouracil/nedaplatin, docetaxel/5-fluorouracil/nedaplatin, vinorelbine+cisplatin, pemetrexed/nedaplatin, vinorelbine/S-1, or S-1 monotherapy, as per the NCCN guidelines [12].

### 2.4. Follow-Up

The first follow-up visit was 2-3 months after treatment. Additional follow-up was offered every 3-4 months for the first two years and every 6-12 months thereafter. Follow-up was ended in August 2019.

### 2.5. Observational Outcomes

For basic information, sex, age, tumor location, T and N stages, and clinical stage were recorded. TNM stages were all restaged according to the 8^th^ edition of the AJCC TNM classification. For treatment-related characteristics, chemotherapy regimens, combined with Endostar or not, numbers of induction chemotherapy cycles, and radiation doses were recorded.

Tumor response and acute adverse events after treatment were followed and recorded. Complete response (CR), partial response (PR), stable disease (SD), and progressive disease (PD) were evaluated by CT scan and endoscopy, according to RECIST 1.1 [14]. CR: all target lesions disappeared. PR: the total diameter of all target lesions is reduced by ≥30%. PD: the total diameter of all target lesions is increased by ≥20%. SD: all target lesions did not reach PR, and the increase did not reach PD. Objective response rate (ORR) = CR + PR. Disease control rate (DCR) = CR + PR + SD.

Adverse events mainly included hematologic toxicity, heart damage, esophagitis, pneumonitis, and skin damage and were graded according to the National Cancer Institute Common Terminology Criteria for Adverse Events (NCI CTCAE) version 3.0 [15].

Locoregional failure was defined as a relapse/progression of the primary tumor or regional lymph nodes. Distant failure was defined as tumor metastasis to distant sites. Any occurrence of this condition during follow-up was considered a failure.

OS and PFS were recorded. OS was defined as the time from treatment initiation to death or loss to follow-up or end of follow-up. PFS was defined as the time from treatment initiation to disease progression (including locoregional failure and distant failure), loss to follow-up, or end of follow-up. Locoregional failure-free survival (LRFFS) was defined as the time from treatment initiation to locoregional failure, loss to follow-up, or end of follow-up.

### 2.6. Statistical Analysis

SPSS 19.0 (IBM, Armonk, NY, USA) was used for statistical analysis. Continuous variables are presented as medians (range). Categorical variables are reported as frequencies (%). OS, PFS, and LRFFS were shown according to the Kaplan-Meier method, and subgroup analyses were conducted using the log-rank test. *P* values <0.05 were considered statistically significant.

## 3. Results

### 3.1. Characteristics of the Patients

Twenty-six patients were included and analyzed. The median age was 58.5 (range, 39-81) years, 21 (80.8%) patients were male, and five (19.2%) were female. Twenty-three (88.5%) patients were scheduled for induction chemotherapy, and all patients received at least one cycle of concurrent chemotherapy. The characteristics of the patients are shown in Table 2.

### 3.2. Treatment Effect

Median follow-up was 31 (range, 4.3-51.3) months for all patients and 40.4 (range, 30.6-51.3) months for survivors. All patients completed radiotherapy without any interruption longer than 7 days. Treatment characteristics are shown in Table 3. Sixteen (61.5%) patients had CR, four (15.4%) achieved PR, one (3.8%) had SD, two (7.7%) developed PD, and three (11.5%) were not evaluable due to missing data. The ORR was 76.9%, and the DCR was 80.8% (Table 4).

### 3.3. Survival

The median PFS and OS were not reached when the present analyses were performed. The 1-, 2-, and 3-year PFS rates were 91.3%, 68.5%, and 63.9%, respectively. The 1-, 2-, and 3-year OS rates were 92.3%, 75.4%, and 71.0%, respectively. The 1-, 2-, and 3-year LRFFS rates were 96.2%, 73.3%, and 73.3%, respectively. The 4-year PFS was 63.9%, the 4-year LRFFS rate was 73.3%, and the 4-year OS was 71.0%, indicating stable survival from 3 to 4 years in those patients (Figures 2(a)–2(c)). The patients with recurrence underwent systemic treatment based on their supervising physicians; they did not undergo further irradiation therapy.

Subgroup analyses were performed, and the results are shown in Table 5 and Figures 2(d)–2(f). The results show that male sex was associated with a poorer 3-year PFS (*P* = 0.034 vs. female sex), middle-thoracic tumor localization was associated with a poorer 3-year OS (*P* < 0.001 vs. the other localizations), and clinical stage III was associated with a poorer 3-year OS (*P* = 0.010 vs. stage IV).

### 3.4. Failure Pattern Analysis

Six (23.1%) patients experienced locoregional failure. Five (19.2%) patients had only locoregional failure, and one (3.8%) had both locoregional and distant failure. Four patients failed at the primary site, and two patients failed in the regional lymph nodes. Three patients developed distant metastases: bone (*n* = 2) and liver (*n* = 1).

### 3.5. Adverse Events

Toxicities related to treatments are summarized in Table 6. No patients developed radiation-related heart or skin damage. Sixteen (61.5%) patients developed grade 1-2 hematologic toxicity, and seven (26.9%) developed grade 3-4 hematologic toxicity. Grade 1-2 radiation-related esophagitis was observed in 15 (57.7%) patients, and grade 3-4 radiation-related esophagitis was observed in one (4.5%) patient. Grade 1-2 radiation-related pneumonitis was observed in 12 (46.2%) patients, and grade 3-4 radiation-related pneumonitis was observed in one (4.5%) patient. No patients died of radiation-related toxicities.

## 4. Discussion

According to an expert consensus [13] and NCCN guidelines [12], the GTV should include the primary tumor and involved regional lymph nodes based on CT images, clinical information, and PET-CT images. CTV should be 3-4 cm above and 3-4 cm below the edge of the GTV. The nodal CTV should expand by 0.5-1 cm from the nodal GTV. For distal esophageal or gastroesophageal junction cancer, in order to reduce the radiation volume to the stomach and other organs, a margin of 2 cm below the GTV edge is acceptable. The radial border should be 1 cm from the outer wall of the esophagus. If the GTV covers essential organs such as the heart and liver, the CTV expansion should be limited to 0.5 cm. For regional nodal volumes, the CTV should be contoured according to the location of the tumor. For distal tumors approaching or involving the gastroesophageal junction, the CTV should cover the celiac, para-aortic, and gastrohepatic lymph nodes. For tumors above the carina, bilateral supraclavicular nodal areas should be included in the CTV, and the recommended borders are to level IV lymph nodes in head and neck cancer [16]. The lower paratracheal nodal stations and upper paratracheal nodal stations and prevascular nodal stations, which correspond to IASLC levels 2, 4, and 3, respectively [17], should also be included. Base on the NCCN guideline, the recommended dose of definitive radiation is 50-50.4 Gy (1.8-2.0 Gy/d) [12].

Nevertheless, when using those treatment parameters, the prognosis of unresectable esophageal cancer is still poor. The 5-year survival is about 25%, and the local recurrence rate is about 40-60% after definitive CRT [5, 6, 18]. The 1- and 3-year overall survival rates are 65% and 28%, respectively [18]. The main failure pattern of definitive CRT is a locoregional failure. The long-term locoregional control rate is 38%-55%, and the predominant site of failure is the primary tumor area [18]. Locoregional failure as the first failure is more common than distant failure [5, 6, 9, 18, 19]. Locoregional failure is the main failure pattern for ESCC who received definitive radiotherapy. About 40%-50% of patients experience locoregional failure [6, 20]. In patients who received selective nodal irradiation, primary tumor recurrence is the main failure pattern [21]. Among all the local failures, 90% of failures are in the GTV, 23% are in the CTV, and 14% are in the PTV; 72% of the patients have failure only in the GTV [9].

Therefore, those data suggest that intensifying local therapy may improve the prognosis of esophageal cancer. Previous studies also demonstrated that a minimum of 65-70 Gy would be needed to achieve tumor control for solid tumors [22]. On the other hand, increasing the radiation dose to esophageal cancer will also increase the dose to the lung, which will increase the risk of severe radiation pneumonitis. Thus, at our center, the target volume definition was modified so that the dose to the tumor could be increased while protecting the lungs at the same time.

Pathological analysis showed that in ESCC, the mean microscopic spread longitudinally beyond the gross tumor is about 10 mm, and 94%-97% of the cases are within 30 mm [23]. Therefore, the CTV1 was defined as 3 cm above and below the edge of the GTVt. Both this area and the primary tumor site have a high risk of relapse because the traditional dose of primary tumor and CTV1 is about 50 Gy, which is not a definitive dose. Thus, the dose to the primary tumor and CTV1 was increased to achieve better locoregional control. In the INT0123 trial, the locoregional control was not improved though the dose of GTV was increased to 64.8 Gy, with 1.8 Gy/day [6]. The INTG0123 trial was carried out using two-dimensional radiotherapy (2DRT), while three-dimensional and IMRT are widely used nowadays. In the present study, the IMRT technique was used, and the dose was increased to 66-68 Gy, with fraction of 2.0-2.2 Gy/day. The biologically effective dose (BED) was about 72-73 Gy, which is a definitive dose for solid tumors [22]. Because of the high dose in the GTV and CTV1, the V20 of the lungs would be very high if the CTV1 was expanded by 0.5-1.5 cm around the esophageal wall. Thus, the CTV1 expansion was limited to 1-2 mm around the esophageal wall.

In terms of toxicity, hematological toxicity was the most common toxicity and was due to chemotherapy. Regarding radiation toxicity, only one patient developed grade 3-4 radiation pneumonitis, and one patient developed grade 3-4 radiation esophagitis. No patients died of toxicity. In the RTOG 8501 trial, the patients who received chemoradiotherapy had more adverse effects than those who received radiotherapy alone, and 10% had life-threatening toxic effects [5]. The INT0123 trial reported that higher radiotherapy doses were related to higher rates of radiation-related deaths [6]. Such toxicity was not observed in the present study, possibly because of the reduced treatment volumes, but this will have to be confirmed in future trials.

Radiation resistance is also an important factor that will impair the effect of radiotherapy. Tumor hypoxia is one of the factors that contribute to radiation resistance [24]. With defects in the endothelium and other structures, blood vessels in tumors are usually structurally and functionally abnormal [25]. These abnormal blood vessels impair the supply of oxygen and results in radiation resistance [26, 27]. Endostar is a recombinant human endostatin that targets new capillary endothelial cells around tumors [28]. Endostar shows an antitumor effect when it is used together with chemotherapy [28–30]. An in vitro study showed that Endostar inhibits the VEGF signal pathways and thus increases the efficacy of radiotherapy [31]. In the present study, patients treated with Endostar combined with CRT showed a trend towards a survival benefit. Still, no significant difference was observed, possibly because of the small sample size. Future trials should also specifically examine this point.

Middle-thoracic tumor localization was associated with a poor OS. This could be related to Endostar. The numbers of patients with cervical, upper thoracic, middle thoracic, and lower-thoracic tumor localization and who received Endostar are 3 (75%), 5 (62.5%), 5 (45.5%), and 1 (33.3%), respectively. Therefore, the proportion of patients receiving Endostar in the middle-thoracic tumor subgroup was low, contributing to a poorer OS. Although the proportion was low in lower-thoracic tumors as well, there were only three patients in this subgroup, and the sample size was too small to draw any definite conclusion. Furthermore, stage III patients had poorer survival than stage IV patients. The small sample size and the use of Endostar could also explain this paradoxical result. In stage III patients, 7/15 (46.7%) received Endostar, while in stage IV patients, 6/8 (75%) received Endostar. This might contribute to a better OS in stage IV patients. According to the subgroup analysis, patients receiving Endostar tended to have better 3-year LRFFS, PFS, and OS, although no statistically significant difference was observed. Future large sample size studies should verify this analysis.

There are some limitations to this study. First, tumor responses were evaluated by CT scan and endoscopy rather than pathological examination. CT is a poor diagnostic tool to evaluate the tumor response in patients after CRT [32]. Second, the number of patients in this study was not enough to draw any firm conclusions. Third, this is a retrospective analysis, and recall bias may exist. Finally, the observation period is short.

## 5. Conclusion

In conclusion, the modified target volume definition and increased dose of definitive chemoradiotherapy in patients with ESCC had low toxicity and might improve survival, but additional trials are necessary to prove the superiority of this strategy.

## Figures and Tables

**Figure 1:** Definition of target volumes. Primary tumor gross tumor volume (GTVt) is shown as the red line. The involved regional lymph node gross tumor volume (GTVnd) is shown as the orange line. The clinical tumor volume (CTV1) is shown as a pink line. The clinical tumor volume for regional nodal volume (CTV2) is shown as the blue line. The planning gross target volume (PGTVt), planning gross tumor volume of lymph nodes (PGTVnd), planning clinical tumor volume (PTV1), and planning clinical tumor volume for regional nodal volume (PTV2) were a 0.5-centimeter expansion from GTVt, GTVnd, CTV1, and CTV2 (PTVs were not shown).

**Figure 2:** (a–c) Kaplan-Meier survival curves for progression-free survival (PFS), overall survival (OS), and locoregional failure-free survival (LRFFS) curves. (d–f) Subgroup survival curves. (d) The overall survival (OS) of the clinical-stage IV subgroup was longer than that of the stage III subgroup (*P* = 0.010). (e) The progression-free survival (PFS) of female patients was longer than that of males (*P* = 0.034). (f) The OS of the middle-thoracic subgroup was shorter than that of the other subgroups (*P* < 0.001).

**Table 1:** Target volume definitions.

	NCCN guideline definition^#^	Modified definition	Prescription dose
GTV	Primary tumor (GTVt) and involved lymph node (GTVnd)	Primary tumor (GTVt) and involved lymph node (GTVnd)	66-68 Gy, 2.0-2.2 Gy/fraction

CTV	3-4 cm expansion above and below the edge of GTVt and 1 cm expansion around the esophageal wall as primary tumor CTV. The nodal GTV plus an expansion of 0.5-1.5 cm as the nodal CTV. Elective nodal regions should be included.	3 cm expansion above and below the edge of the GTVt and 1-2 mm expansion around the esophageal wall as CTV1. Elective nodal regions defined as CTV2 and GTVnd should include in CTV2.	CTV1: 66-68 Gy, 2.0-2.2 Gy/fraction;CTV2: 46 Gy, 2.0 Gy/fraction

PTV	0.5-1 cm expansion	0.5 cm expansion	

^#^Esophageal and esophagogastric junction cancers, V2.2019.

**Table 2:** Characteristics of the patients.

Characteristics, *n* (%)		Patients (*n* = 26)
Sex	Male	21 (80.8)
	Female	5 (19.2)

Age (years)	≥75	3 (11.5)
	<75	23 (88.5)

Tumor localization	Cervical	4 (15.4)
	Upper thoracic	8 (30.8)
	Middle thoracic	11 (42.3)
	Lower thoracic	3 (11.5)

T stage	1	0
	2	2 (8.7)
	3	8 (30.8)
	4	13 (50.0)
	x	3 (11.5)

N stage	N0	0
	N+	26 (100)

Clinical stage	IIB	2 (8.7)
	III	15 (57.7)
	IV	8 (30.8)
	X	1 (3.8)

**Table 3:** Characteristics of the treatments.

Characteristics		Patients (*n* = 26)
Chemotherapy regimens, *n* (%)	TP^#^	20 (76.9)
	Others^∗^	6 (23.1)

Combine with Endostar, *n* (%)	Yes	14 (53.8)
	No	12 (46.2)

Number of induction chemotherapy cycles, *n* (%)	0	3 (11.5)
	1	4 (15.4)
	2	16 (61.5)
	≥3	3 (11.5)

Radiation therapy, *n* (%)	One-stage strategy	13 (50)
	Two-stage strategy	13 (50)

Radiation dose (cGy)	Median (range)	6800 (6620-6930)
	>6800, *n* (%)	7 (26.9)
	≤6800, *n* (%)	19 (73.1)

^#^TP, paclitaxel+nedaplatin. ^∗^Other chemotherapy regimens included TPF (paclitaxel+nedaplatin+S-1, *n* = 1); DPF (docetaxel+nedaplatin+S-1, *n* = 1); NP (vinorelbine+cisplatin, *n* = 1); PP (pemetrexed+nedaplatin, *n* = 1); vinorelbine+S-1, *n* = 1; S-1 monotherapy, *n* = 1.

**Table 4:** Tumor response assessment^∗^.

Clinical stage	All (*n* = 26)	IIB (*n* = 2)	III (*n* = 15)	IV (*n* = 8)	X (*n* = 1)
CR	16	1	8	7	0
PR	4	0	3	1	0
SD	1	0	1	0	0
PD	2	0	1	0	1
Not evaluable	3	1	2	0	0
ORR (%)	76.9	50	73.3	100	0
DCR (%)	80.8	50	80.0	100	0

^∗^According to CT scan and endoscopy. CR: complete remission; PR: partial remission; SD: stable disease; PD: progression disease; objective response rate (ORR) = CR + PR; disease control rate (DCR) = CR + PR + SD.

**Table 5:** Subgroup analysis for the survival of the patients.

Characteristics		*N* (%)	3 y LRFFS		3 y PFS		3 y OS	
			%	*P*	%	*P*	%	*P*
Sex	Male	21 (80.8)	63.6	0.051	57.9	0.034	68.4	0.530
	Female	5 (19.2)	100		100		80	

Age (years)	≥75	3 (11.5)	66.7	0.771	67.1	0.862	76.5	0.069
	<75	23 (88.5)	50.0		50.0		33.3	

Tumor localization	Cervical	4 (15.4)	66.7	0.059	66.7	0.064	100	<0.001
	Upper thoracic	8 (30.8)	85.7		85.7		100	
	Middle thoracic	11 (42.3)	46.8		46.8		36.4	
	Lower thoracic	3 (11.5)	66.7		66.7		100	

T stage	3	8 (38.1.)	85.7	0.202	68.6	0.895	72.9	0.927
	4	13 (61.9)	73.8		73.8		75.5	

Clinical stage	III	15 (65.2)	60.3	0.067	60.3	0.067	63.8	0.010
	IV	8 (34.8)	83.3		85.7		100	

Combined with Endostar	Yes	14 (53.8)	71.4	0.849	64.3	0.400	78.6	0.201
	No	12 (46.2)	68.8		53.5		61.1	

LRFFS: locoregional failure-free survival; PFS: progression-free survival; OS: overall survival.

**Table 6:** Treatment-related adverse events.

Adverse events, *n* (%)	Grade 0	Grade 1-2	Grade 3-4
Hematologic toxicity	3 (11.5)	16 (61.5)	7 (26.9)
Heart damage	26 (100)	0	0
Esophagitis	10 (38.5)	15 (57.7)	1 (4.5)
Pneumonitis	13 (50.0)	12 (46.2)	1 (4.5)
Skin damage	26 (100)	0	0

## Data Availability

The datasets used and/or analyzed during the current study are available from the corresponding authors on reasonable request.

## Abbreviations

ESCC: Esophageal squamous cell carcinoma
PGTV: Planning gross tumor volume
PTV1: Planning clinical tumor volume
PFS: Progression-free survival
OS: Overall survival
LRFFS: Locoregional failure-free survival
IMRT: Intensity-modulated radiation therapy
3DCRT: Three-dimensional radiation
GTV: Gross tumor volume
CTV: Clinical target volume
GTVt: Primary tumor
GTVnd: Involved lymph node
PGTVt: Planning gross target volume
PGTVnd: Planning gross tumor volume of lymph nodes
PTV2: Planning target volumes of CTV2
CR: Complete response
PR: Partial response
SD: Stable disease
PD: Progressive disease
ORR: Objective response rate
DCR: Disease control rate
NCI CTCAE: National Cancer Institute Common Terminology Criteria for Adverse Events
2DRT: Two-dimensional radiotherapy.
